# Exploration of gene functions for esophageal squamous cell carcinoma using network-based guilt by association principle

**DOI:** 10.1590/1414-431X20186801

**Published:** 2018-04-19

**Authors:** Wei Wu, Bo Huang, Yan Yan, Zhi-Qiang Zhong

**Affiliations:** 1 Department of Gastroenterology (40th Ward), Daqing Oilfield General Hospital, Daqing, China; 2 Department of Ultrasonics, Daqing Oilfield General Hospital, Daqing, China

**Keywords:** Esophageal squamous cell carcinoma, Gene oncology, Guilt by association, Differentially expressed genes, Area under the curve

## Abstract

Gene networks have been broadly used to predict gene functions based on guilt by association (GBA) principle. Thus, in order to better understand the molecular mechanisms of esophageal squamous cell carcinoma (ESCC), our study was designed to use a network-based GBA method to identify the optimal gene functions for ESCC. To identify genomic bio-signatures for ESCC, microarray data of GSE20347 were first downloaded from a public functional genomics data repository of Gene Expression Omnibus database. Then, differentially expressed genes (DEGs) between ESCC patients and controls were identified using the LIMMA method. Afterwards, construction of differential co-expression network (DCN) was performed relying on DEGs, followed by gene ontology (GO) enrichment analysis based on a known confirmed database and DEGs. Eventually, the optimal gene functions were predicted using GBA algorithm based on the area under the curve (AUC) for each GO term. Overall, 43 DEGs and 67 GO terms were gained for subsequent analysis. GBA predictions demonstrated that 13 GO functions with AUC>0.7 had a good classification ability. Significantly, 6 out of 13 GO terms yielded AUC>0.8, which were determined as the optimal gene functions. Interestingly, there were two GO categories with AUC>0.9, which included cell cycle checkpoint (AUC=0.91648), and mitotic sister chromatid segregation (AUC=0.91597). Our findings highlight the clinical implications of cell cycle checkpoint and mitotic sister chromatid segregation in ESCC progression and provide the molecular foundation for developing therapeutic targets.

## Introduction

Esophageal squamous cell carcinoma (ESCC), one of the most lethal malignancies in humans, results in more than 400,000 deaths per year. Patients with ESCC are usually diagnosed at an advanced stage, and the 5-year survival rate is reported to be less than 15% (1). Early diagnosis has been the only promising means of achieving better outcomes, and no reliable diagnostic marker for ESCC has been found. Thus, identifying non-invasive biomarkers to assist in the diagnosis of ESCC in clinical settings is urgently needed.

ESCC development is influenced by multiple factors, involving changes of gene expression as well as physiological structure (2). With the rapid development of molecular biology, many scholars have conducted in-depth analysis on the etio-pathogenesis of ESCC from gene level, and a large number of significant genes has been detected. For instance, up-regulation of epidermal growth factor receptor and cyclin D1, and expression of p53 mis-sense mutations have been associated with ESCC progression (3). Recent high-throughput cancer genome sequencing revealed several gene mutations (ADAM29, MLL2, ASH1L, SETD1B, MLL3, EP300, CREBBP, and FAM135B) in ESCC (4). Nevertheless, the mechanism of ESCC has not been fully elucidated. Therefore, further studies are imperative to understand the underlying molecular basis of ESCC.

Microarray analysis has been broadly used to identify the potential targets in ESCC. Therefore, investigators have employed bioinformatics methods to study the microarray profiles of ESCC and explore molecular mechanism underlying ESCC. GSE20347 is one of the microarray profiles of ESCC deposited by Nan et al. (5), who studied the copy number changes and the relationship to gene expression in ESCC. In 2014, using the same data deposited by Nan et al. (5), Li et al. (6) identified 33 differentially expressed miRNAs and 1322 differentially expressed genes (DEGs) with a close relationship with ESCC. Moreover, Tung et al. (7) used the same dataset and found that RUVBL1 and CNIH could be useful biomarkers for discriminating cancer from normal tissues in Taiwanese ESCC patients. However, research related to the genetics of ESCC has paid attention to a single gene or a single miRNA.

To a certain degree, function-based analyses are better in producing more reproducible results, relative to individual gene-based methods (8). Of note, understanding gene function is a central challenge of biology (9). Characterizing gene function is a complicated task, partially because biological functions contain the integrated activities of many genes. Moreover, the same gene may have diverse functions relying on different context. Despite the importance of comprehending gene function, little attention has been paid to multifunctionality (MF) in the functional genomics literature. Previously, the attributes of genes were considered to be associated with MF intuitively (for example, pleiotropy as well as hubness), yet these were seldom discussed in the setting of MF. Although close to MF in definition, pleiotropy is not typically applied to refer exclusively to molecular traits and is frequently referred to the effect of mutation on phenotype. The high connectivity of hubs is usually regarded to reflect biological “importance” (10). Conversely, MF is defined with reference to genes possessing multiple molecular functions, each of which can be characterized by the gene set (the corresponding products) inferred to be interacted in a particular biological setting. Moreover, Gillis et al. (11) have demonstrated that MF is a primary driver for predicting gene functions.

A general approach to describe and assess function based on computational technique is important. One of the broadly used methods for expounding the functions of un-annotated genes, that is to say, for gene function prediction, is the guilt-by-association (GBA) principle (12). The GBA principle claims that genes participating in the same cellular processes tend to have similar properties, which allows to statistically infer previously unknown functions of a gene relying on the prior knowledge about other genes and association data (13). GBA has been indicated to predict gene function in various types of biological networks, for example, gene co-expression network (14). Genetic factors can disturb protein levels, thereby disturbing molecule interactions. The characterization of networks clarifies the complicated interactions and interwoven relationships, which control cellular functions (15). Understanding the networks will offer novel insights to reveal the molecular pathogenesis of ESCC.

In our analysis, we planned to detect disease-associated gene functions in ESCC and to obtain more insight into the mechanisms underlying ESCC. In order to achieve this goal, we utilized the network-based GBA principle, comprising the following steps: identifying DEGs between the two groups; constructing the differentially co-expressed network (DCN) relying on DEGs, followed by recruiting GO annotations based on the known database and DEGs; and identifying gene functions using GBA principle on the basis of area under the receiver operating characteristics curve (AUC). GO terms with AUC>0.8 were defined as the optimal gene functions for ESCC patients.

## Material and Methods

### Microarray data

To identify genomic bio-signatures for ESCC, microarray dataset of GSE20347 (5) was downloaded from a public functional genomics data repository of Gene Expression Omnibus (GEO) database. GSE20347 was conducted on the Affymetrix (USA) Human U133A platforms (GPL571), which consisted of expression profiles of 17 pairs of ESCC tissues and matched normal adjacent tissues from Taiwanese male patients in China. Annotation information file for all probe sets (ATH1, genome array developed by Affymetrix) was obtained from the R package. The probe annotations and the primary files were extracted for further analysis.

### Data preprocessing

Data analysis started by processing a set of signal intensity files for Affymetrix expression arrays (CEL). The probe-level data in CEL style were transformed into expression profiles. Next, for any missing values of probe (NA or the probes with expression value of 0), we imputed missing data using k-nearest neighbor algorithm (16). Robust multiarray average (17) was used to implement background correction and quantile normalization. Finally, probes set-level information was mapped to the genomics to further obtain the gene symbols based on the package annotation (18). Totally, 12.436 genes were identified for subsequent analysis.

### Analysis of DEGs

DEGs between matched normal adjacent and ESCC tissues were first extracted using the paired *t*-test available at LIMMA package (19). After that, to circumvent the multi-test problem, which might result in too many false positive results, Benjamin and Hochberg correction was applied to correct the raw P-values into false discovery rate (FDR) (20). Only those genes with FDR<0.001 and |log fold change (FC)|>2 were regarded as differentially expressed between the two groups.

### DCN construction

Cytoscape (http://cytoscape.org/), an open-source software, can combine molecular interactions with microarray expression profile into a unified network. Hence, we inputted DEGs into the Cytoscape tool to show the structure of DEGs relationships. Further, in an attempt to evaluate the co-expressed strength of every interaction within the DEG-based network, Spearman correlation coefficient (SCC), which measured the strength of association of two variables, was employed in this work, which could assess the co-expression probability of two variables by measuring the strength of association of two co-expressed variables and whose range is from -1 to 1 inclusively (21). The weight value of one interaction was defined as the SCC absolute value of the corresponding edge; greater weight values indicated that the interaction was more relevant to the given disease.

### GO annotations

GO consortium (http://geneontology.org/), a community-based bioinformatics database, offers gene function information (22). First, human GO annotations including 19,003 functions with 18,402 genes were obtained from GO consortium. As known, biological functions having few genes might not have sufficient biological information, but gene functions with too many genes might be too generic (23). Previous studies have filtered GO terms by size such that each remaining term had between 20 and 1000 associated genes, a range that generally gives stable performance (11,24). In our study, to receive stable performance, a set of GO groups excluding the GO terms with less than 20 genes or more than 1000 genes were reserved, and the subset of GO annotations having between 20 and 1000 associated genes was assessed. We defined these GO annotations having between 20 and 1000 associated genes as the seed GO terms. Then, to assess the association of these GO terms with ESCC, we aligned the identified DEGs above the subset of seed GO terms. If a seed GO term had less than 20 DEGs, it would be discarded. Therefore, only GO categories covering ≥20 DEGs were retained for subsequent analysis.

### Predicting gene functions using GBA method

Gene networks can be broadly applied to infer the gene functional relationships based on the GBA principle. Herein, we used GBA method to predict significant gene-associated GO terms involved in the ESCC progression by means of three-fold cross-validation to identify a sorted list of scoring genes in the DCN as to how they belonged in the known gene function. The sum of co-expression values between the training set (co-expression) and the candidate gene was divided by the sum of co-expression values between the genes outside the training set and the candidate gene to analyze degree of candidacy. In detail, for each gene in the DCN, the MF score in the given GO term was calculated based on the formula described in the study by Gillis and Pavlidis (11).

AUC is a measure used to assess the predictive ability of machine learners in support vector machines (SVM) model (25). Thus, in our study, based on SVM, AUC was computed to further evaluate the classification abilities between ESCC and control samples. The AUC scores were ranked from the highest to the lowest and the ranks of GO terms were sorted oppositely. The AUC of 0.5 represents the classification at chance levels, while the AUC of 1.0 is a perfect classification. Based on the literature, an AUC greater than 0.7 is considered good (24). In our study, GO terms with AUC>0.8 were identified and regarded as the optimal gene functions.

## Results

### Analysis of DEGs and DCN construction

The expression profiles before and after normalization are exhibited in Figure 1A and B.

**Figure 1.** *A*, Box plot of gene expressions in esophageal squamous cell carcinoma (ESCC) and the matched normal adjacent samples before normalization. *B*, Box plot of gene expressions in ESCC and matched normal adjacent samples after normalization. The X-axis indicates samples and the Y-axis is expression level of genes. The black line in the center is the median expression value; the consistent distribution represented a good standardization.

To obtain DEGs, we downloaded publicly available microarray data GSE20347 from the GEO database. Following data pretreatment, a total of 43 genes were identified as DEGs at FDR<0.001 and |logFC|>2. The list of DEGs is shown in Table 1. The most significant 10 DEGs were HOXB7 (FDR=1.69E-07), SMYD3 (FDR=2.36E-07), ECT2 (FDR=3.19E-07), CBX3 (FDR=4.69E-07), AURKA (FDR=7.46E-07), WDHD1 (FDR=9.01E-07), MTHFD2 (FDR=2.87E-06), KIF4A (FDR=5.72E-06), DUSP12 (FDR=5.94E-06), and FNDC3B (FDR=6.18E-06).

**Table 1.** List of differentially expressed genes (DEGs)

Genes	|log FC)|	FDR
HOXB7	2.058	1.69E-07
SMYD3	2.237	2.36E-07
ECT2	5.174	3.19E-07
CBX3	3.540	4.69E-07
AURKA	2.981	7.46E-07
WDHD1	3.398	9.01E-07
MTHFD2	3.201	2.87E-06
KIF4A	2.436	5.72E-06
DUSP12	3.427	5.94E-06
FNDC3B	2.085	6.18E-06
RFC4	2.147	6.29E-06
HJURP	2.969	6.51E-06
SERPINH1	3.521	6.53E-06
RAD51	2.885	6.70E-06
FZD2	3.203	6.98E-06
MFAP2	3.131	7.10E-06
LPCAT1	2.765	8.08E-06
HMGB3	2.120	8.38E-06
FOXM1	2.641	8.82E-06
TRAM2	2.599	9.10E-06
GTF2E1	2.078	9.16E-06
NEMP1	3.884	9.29E-05
SNAI2	3.645	9.31E-06
FSCN1	2.073	9.45E-06
DNMT3B	2.098	9.79E-06
RUVBL1	2.263	1.72E-05
SLC39A14	2.006	1.79E-05
PPT1	2.214	1.82E-05
TOP2A	2.784	2.12E-05
MYO5A	2.393	3.73E-05
UMPS	2.261	3.93E-05
MINPP1	2.078	3.96E-05
SPAG5	2.317	4.06E-05
SLC39A6	2.463	4.11E-05
KPNA2	2.060	4.45E-05
THAP12	2.671	6.25E-05
CERS2	3.065	8.44E-05
PLOD3	2.821	9.61E-05
PTDSS1	2.257	9.98E-05
ACD	2.042	1.00E-04
C20orf27	2.826	2.89E-04
E2F6	2.111	3.06E-04
CALU	2.383	3.17E-04

FC: Fold change; FDR: False discovery rate.

To further reveal the biological activities of DEGs, a DCN with 43 nodes and 919 interactions for ESCC is displayed using Cytoscape (Figure 2), which suggested that all DEGs were aligned to the DCN. The interacted strength was an index used to assess the interactions in the DCN. As a result, the weight values were assigned to each edge based on SCC. The weight scores were different among interactions. The interactions having greater weight scores might be more important for ESCC than the others. The weight distribution of the interactions in the DCN is listed in Figure 3. The majority of interactions were distributed in the weight range of 0.4–0.5 (380 interactions, 41.35%), followed by the range between >0.5–0.6 (232 interactions, 25.24%), >0.6–0.7 (168 interactions, 18.28%), >0.7–0.8 (84 interactions, 9.14%), >0.8–0.9 (30 interactions, 3.26%), and >0.9–1.0 (25 interactions, 2.72%). Of note, the interaction of KIF4A and TOP2A provided the highest weight value of 0.999834. The interaction of SPAG5 and TOP2A had the second higher weight value of 0.999832.

**Figure 2.** Differentially co-expressed network construction for esophageal squamous cell carcinoma based on differentially expressed genes.

**Figure 3.** Pie chart showing the weight distribution of interactions in the differential co-expression network. The weight values were classified into the following groups: >0.9–1.0, >0.8–0.9, >0.7–0.8, >0.6–0.7, >0.5–0.6 and 0.4–0.5.

### Collecting GO annotations

In order to identify significant GO categories, 19,003 GO terms covering 18,402 genes were firstly collected from the GO Consortium. After discarding several GO terms with gene size of <20 or >1000, 1755 seed GO gene sets remained in our analysis. Then, the functions having DGEs <20 were removed, and 67 informative GO terms involved in 43 DEGs were reserved.

### Predicting gene functions and identifying the optimal gene functions

Based on the combination of GO terms and DCN, we predicted the gene-related GO terms using the GBA method. Firstly, for each gene in a GO term, we counted the MF score, which affected the counting membership in a GO category by how much the gene contributed to that given GO term. The greater the MF score of a gene, the greater the extent to which it ought to a good candidate for a given function. Thus, a single ranked list of genes that best captured candidacy across all functions was equivalent to a list of genes sorted by MF scores. The specific MF distribution for DEGs in 67 informative GO terms are shown in Table 2. The top 5 genes with the higher MF scores were SNAI2 (MF=0.000834), KIF4A (MF=0.000778), ECT2 (MF=0.000756), MYO5A (MF=0.000743), and TOP2A (MF=0.000552).

**Table 2.** Distribution of multifunctionality (MF) score of differentially expressed genes.

Genes	MF scores
SNAI2	0.000834
KIF4A	0.000778
ECT2	0.000756
MYO5A	0.000743
TOP2A	0.000552
RAD51	0.000498
AURKA	0.000443
SMYD3	0.000436
RUVBL1	0.000428
PPT1	0.000417
DNMT3B	0.000388
FZD2	0.000358
LPCAT1	0.000269
RFC4	0.000253
SERPINH1	0.000246
FOXM1	0.000239
ACD	0.000200
UMPS	0.000194
PLOD3	0.000194
SLC39A6	0.000191
HJURP	0.000190
SLC39A14	0.000182
SPAG5	0.000179
KPNA2	0.000127
MTHFD2	0.000123
CBX3	0.000111
FNDC3B	0.000104
HOXB7	9.81E-05
PTDSS1	9.77E-05
FSCN1	9.74E-05
DUSP12	8.57E-05
CALU	8.46E-05
E2F6	7.00E-05
CERS2	6.43E-05
HMGB3	5.01E-05
MFAP2	4.49E-05
MINPP1	4.07E-05
GTF2E1	4.02E-05
WDHD1	3.62E-05
TRAM2	2.81E-05
NEMP1	0
THAP12	0
C20orf27	0

Intuitively, if one wanted to select a single ranking, the gene owning the most significant GO categories could be predicted as being in all GO terms. This is because if one gene was enriched in 100 GO terms (highest MF score) and another gene was involved in only one (lowest MF score), by placing the former gene ahead of the latter gene in a fixed ranking, we frequently made a correct prediction across all GO categories. Consequently, we implemented 3-fold cross-validation on MF scores to compute AUC for GO terms, aiming to distinguish ESCC from controls.

The AUC distribution for GO categories is illustrated in Figure 4. From this figure, we observe that the AUC for GO terms ranged from 0.3 to 0.9, and the frequency of GO terms with the AUC of 0.55∼0.65 was higher than that of the other GO terms. If we used it as a predictor of GO category member, we ought to obtain AUC values of over 0.5 for GO terms. Based on AUC>0.7, a total of 13 GO terms were identified. It is noteworthy that 6 out of 13 GO terms had the AUC>0.8 and these 6 GO terms were determined as the optimal gene functions (Table 3). Interestingly, there were two GO categories with AUC>0.9, including cell cycle checkpoint (AUC=0.91648), and mitotic sister chromatid segregation (AUC=0.91597).

**Figure 4.** Gene function prediction by means of guilt by association method based on area under the curve (AUC) values. The histogram shows AUCs across all gene oncology categories, which were identified relying on a single list constructed from the count of co-expression members.

**Table 3.** List of optimal gene functions relying on area under the curve (AUC)>0.8

Gene oncology (GO) terms	AUC	Gene No.
Cell cycle checkpoint	0.91648	39
Mitotic sister chromatid segregation	0.91597	29
Regulation of cyclin-dependent protein serine/threonine kinase activity	0.88779	32
Reproduction	0.84575	23
DNA damage checkpoint	0.84231	26
G1/S transition of mitotic cell cycle	0.84194	34

## Discussion

Currently, gene-related functional investigations seem rewarding in exploring functional insights (26). Unfortunately, investigating gene function is a central challenge of biology. To solve this problem, many techniques have been proposed to extend GBA to connections to identify gene functions (27,28). The GBA principle is the foundation for most gene function prediction approaches, which typically employs relational data (for instance, interactions) to predict gene membership in categories of gene function (29). Generally, network based-GBA analysis may make exhaustive examining issues faster and easier than the simple GBA principle. Further, the combination of gene function prediction and network analysis is sparse. Consequently, we used DCN-based GBA principle to extract the optimal gene functions for ESCC based on GO information as well as gene expression data, thereby further exploring the molecular mechanisms of ESCC. In total, 13 GO categories were obtained relying on AUC>0.7, which indicates a good classification ability. Six out of 13 GO terms having AUC>0.8 were determined as optimal gene functions. Interestingly, there were two GO categories with AUC>0.9, including cell cycle checkpoint and mitotic sister chromatid segregation.

Cell cycle progression is supervised by checkpoint mechanisms, and checkpoints are regarded as the gatekeepers of genome integrity (30,31). A variety of surveillance mechanisms exist in cells to ensure maintenance of genomic stability against various types of damage to the genome. The G1 checkpoint prevents replication of damaged DNA, while genomic integrity before mitosis is monitored by the G2 checkpoint, which promotes G2 arrest on detection of DNA damage. Failure of cell cycle checkpoints results in genomic instability, which predisposes cells to neoplastic transformation and tumor development (32). Moreover, Hu et al. (33) have suggested that inactivation of the cell cycle checkpoint plays important roles in ESCC progression. Thus, the results obtained in our study further support the idea that cell cycle checkpoint is closely associated with ESCC onset and progression.

In the process of mitosis, a crucial step of the cell cycle is the segregation of sister chromatid. Mitotic checkpoints control sister chromosome segregation (34). Abnormalities in double-strand break repair can ultimately cause chromosomal instability as a result of repeated chromosome breakage-fusion-bridge cycles (35). Chromosome segregation is controlled by kinetochores, which guarantee the fidelity of segregation (36). Aberrant function of kinetochores results in losses or gains of large portions of chromosomes (37). Chromosomal instability is distinct in cancer pathogenesis (38). It is worth noting that abnormalities of chromosome segregation exert key functions in promoting tumor formation (39). Above all, the results demonstrate that dysregulation of mitotic sister chromatid segregation endows ESCC development and progression, at least partially, by regulating chromosomal stability.

Although we obtained several significant gene functions in ESCC, there were some limitations in our study. Our study was implemented based on bioinformatics methods but the conclusions have not been tested using animal experiments. Furthermore, the sample size was limited. Thus, more work is warranted to further reveal the molecular basis of ESCC and to apply the molecular detection to the clinical setting.

Despite that our study lacked experimental investigations, our results supported some preliminary evidence to uncover potential candidate therapeutic strategies for ESCC. Our findings demonstrated that using specific blockage-related GO functions in ESCC will provide novel insights for therapeutics and preventive approaches. However, the association between GO terms and ESCC still needs to be tested in animal experiments.
